# Clinical Comparison of Preterm Birth and Spontaneous Preterm Birth in Severe Preeclampsia

**DOI:** 10.1155/2022/1995803

**Published:** 2022-09-15

**Authors:** Yanqing Wen, Xiaoyan Yang

**Affiliations:** Department of Obstetrics and Gynecology, Women and Children's Hospital of Chongqing Medical University, Chongqing, China

## Abstract

Severe preeclampsia is accompanied by many complications, which is extremely harmful to pregnant women and fetuses. However, in the classification of preterm birth, it is generally divided into spontaneous preterm birth and therapeutic preterm birth, and insufficient attention has been paid to preterm birth in severe preeclampsia. This article aims to explore the clinical difference between preterm birth in severe preeclampsia and spontaneous preterm birth. In the experiment, this paper selected pregnant women who delivered and were treated in a hospital from April 2010 to April 2020 as cases. In terms of grouping, not only are they divided into severe eclampsia group (observation group 1), spontaneous preterm birth group (observation group 2), and general delivery group (control group) according to the cause of premature birth, but also according to the gestational age of severe eclampsia onset, preterm weeks, and other groups. Not only the clinical difference between severe preeclampsia preterm birth and spontaneous preterm birth was compared horizontally, but also the factors affecting the complications of preterm pregnant women, perinatal asphyxia rate, and mortality were longitudinally analyzed. The experimental results in this paper showed that there were significant differences in maternal complications and neonatal mortality between the severe preeclampsia preterm group and the spontaneous preterm group (*P* < 0.05). In addition, the severe preeclampsia preterm birth group was more harmful than the spontaneous preterm birth group. The complication rate of the severe preeclampsia preterm birth group was 10% higher than that of the spontaneous preterm birth group, and the neonatal mortality rate was 2% higher.

## 1. Introduction

Fertility is a necessary part of human reproduction and development, but premature birth is also very likely to occur in childbirth, which is very harmful to pregnant women and newborns. The fetal lungs of neonates delivered after 34 weeks of gestation are basically mature, and the incidence of neonatal ventricular asphyxia, hyaline membrane disease, and neonatal hypoxic ischemic encephalopathy after delivery is low. Delivery after 34 weeks of gestation can effectively shorten the length of hospital stay, reduce related treatment costs, and achieve better long-term prognosis. Early treatment for preterm birth can effectively improve the survival rate of neonates, and patients with severe eclampsia are at greater risk, and early prevention is better. Therefore, research on preterm birth and spontaneous preterm birth in severe preeclampsia is necessary.

Spontaneous preterm birth accounts for a large proportion of patients with preterm birth, and many scholars have conducted research on spontaneous preterm birth because of its greater treatability. Campbell studied a rare delayed hypersensitivity reaction called autoimmune progesterone dermatitis in spontaneous preterm labor [1]. Hochwald O assessed the effect of pregnancy interval on subsequent preterm birth rates in women with previous spontaneous preterm birth. He designed a retrospective cohort study with a national longitudinal dataset from the Dutch Perinatal Registry [2]. In his study, Gray C used miRNA arrays to analyze the plasma of healthy women from their first pregnancy at 20 weeks of gestation to analyze spontaneous preterm birth [3]. Rappoport N identified only two intergenic loci associated with PTB at the genome-wide significance level: rs17591250 (*P* = 4.55*E* − 09) on chromosome 1 and rs1979081 (*P* = 3.72 *E *−* *08) on AMR chromosome 8 in the AFR population to judge spontaneous preterm birth [4]. However, related scholars are more focused on the causes of spontaneous preterm birth, and the research on related clinical characteristics is not enough. Severe eclampsia is a serious disease during pregnancy. Because of its greater harm, it is likely to cause greater consequences once it occurs. There are also many prevention studies on it. The Rasmussen S's study found that after preterm delivery in the first pregnancy without preeclampsia, the risk of preterm preeclampsia in the second pregnancy was 4–7 times higher than that after full-term delivery. The risk term of eclampsia is 2–3 times higher in preterm pregnancies than in the term postpartum [5]. Inouye found that acute EBV infection should be included in the differential diagnosis of preeclampsia with severe features. Supportive care and observation can prevent iatrogenic preterm birth [6]. Abe is particularly interested in blood pressure in patients with severe eclampsia, and he has studied the relationship between blood pressure and perinatal growth [7]. Bouchet N studied the relationship between labor cycles and perinatal survival and complications in patients with severe eclampsia [8].

In this study, compared with the cesarean section, women with vaginal delivery will have much fewer complications, especially the symptoms of placental abruption, and vaginal delivery will be much lower than cesarean section. For neonatal asphyxia or mortality, in the presence of severe eclampsia, the neonatal mortality rate of vaginal delivery is higher than that of cesarean section. The innovations of this paper are as follows: in the study, not only the clinical characteristics of the severe preeclampsia preterm birth group and the spontaneous preterm birth group were compared and analyzed, but also the importance of regular physical examination was also studied, which plays an important role in the prevention and treatment of preterm birth in severe preeclampsia.

## 2. Clinical Features of Preterm Birth

### 2.1. Spontaneous Preterm Birth

The methods for predicting preterm birth are also different, especially for the biochemical prediction of preterm birth, which is even more diverse. For example, fFN and serum relaxin in vaginal secretions or cervical mucus are commonly used, and blood and urine routines are tested to observe whether there is obvious infection. Finally, combined with relevant medical history and combined with ultrasound to detect cervical morphological changes and cervical length shortening, it can more accurately predict premature birth, as shown in Figure 1. Schools for pregnant women should be actively carried out, prepregnancy and prenatal education should be popularized, pregnancy examination procedures should be improved, health care during pregnancy should be standardized, and awareness of preventive health care for pregnant women should be raised. Early attention should be paid to appropriate preventive treatment and appropriate medical intervention [9, 10], in order to prolong the gestational age as much as possible, reduce the incidence of preterm birth, improve the survival rate of preterm infants, and improve the quality of life and late prognosis of preterm infants.

As shown in Figure 2, for the treatment of preterm birth, the principle is still to prolong the gestational age as much as possible to gain time for the promotion of fetal lung maturation. In addition to the general proper bed rest, for the choice of drugs to suppress uterine contractions, the method of small doses of magnesium sulfate intravenously combined with oral ritodrine hydrochloride tablets is usually used, which has a good effect. At the same time, it is necessary to gain time to give a single course of dexamethasone intramuscular injection. If infection is clearly present and fetal distress occurs, the pregnancy should be terminated as soon as possible. When the gestational age exceeds 34 weeks, the fetal lungs are basically mature, the neonatal survival rate is significantly increased, the complications are reduced, and the continued pregnancy may increase the risk of infection. Studies have found that those with intrauterine infection have the shortest time to preserve the fetus, and preterm birth is often unavoidable [11, 12]. Also, because of multiple pregnancy and paralyzed uterus, etc., without infection, the pregnancy time is relatively long. Cervical cerclage should be performed at 14–18 weeks of gestation for patients with cervical insufficiency, and attention should be paid to body rest and proper fetal protection after surgery. It can prolong the time of pregnancy, and even reach full term. Late miscarriage or early preterm birth (before 32 weeks of gestation) is likely to occur if it is detected late and intervened late.

### 2.2. Preterm Birth with Severe Preeclampsia

Severe antenatal eclampsia is still an important cause of threatening delivery mothers and newborns. Patients with early-onset severe preeclampsia gradually worsened after 30–32 weeks of gestation. Due to the lack of early specific diagnostic indicators, once clinical symptoms such as edema and proteinuria appear, the disease progresses rapidly and is difficult to control. Iatrogenic preterm birth is often caused by various serious complications [13, 14]. The fetal lungs of severe preeclampsia have the phenomenon of precocious puberty, and the neonatal asphyxia rate and mortality rate of severe preeclampsia cases at 36 weeks of gestation are the lowest. The effects of severe preeclampsia on pregnant women and fetuses are shown in Figure 3.

Severe preeclampsia (SPE) is one of the serious complications of obstetrics, which can cause uteroplacental hypoperfusion, vascular endothelial injury, and release of inflammatory factors, resulting in a series of clinical symptoms. Umbilical artery blood flow, as an effective indicator of placenta-fetal blood flow resistance, plays an important role in the assessment of fetal intrauterine development. In normal pregnancy, the umbilical artery-placental blood flow resistance decreased with the increase of gestational weeks, and the ultrasound showed that the ratio of peak systolic blood flow velocity to end-diastolic blood flow velocity gradually decreased. However, when some factors cause the increase of blood flow resistance in the placenta and umbilical artery, it is manifested as an abnormal increase in S/*D*, and even disappearance or reverse of umbilical artery end-diastolic blood flow (AEDV/REDV). Current studies have shown that abnormal end-diastolic blood flow of the umbilical artery is closely related to perinatal death, intracranial hemorrhage, periventricular leukomalacia, bronchopulmonary hypoplasia, respiratory distress syndrome, necrotizing enteritis, and other neonatal organ system damage. These are among the indicators that suggest a poor intrauterine environment and predict poor perinatal outcomes [15, 16]. Symptoms of preterm women with severe preeclampsia are shown in Figure 4.

Termination of pregnancy is the only effective treatment for early-onset severe preeclampsia [17]. The patient's clinical characteristics, disease status, gestational age, and fetal maturity, and the choice of expected treatment effects should be fully considered: timing and mode of pregnancy. Premature termination of pregnancy may reduce neonatal survival, and prolonged gestational age may increase maternal and fetal mortality. In this study, adverse maternal and perinatal outcomes decreased with increasing gestational age at termination of pregnancy. From a maternal point of view, elective cesarean section carries certain risks. Risks of anesthesia, blood loss and transfusion, and postoperative complications such as thrombotic disease and infection have an impact on patient recovery and fertility and may affect breastfeeding and lead to depression. Therefore, the main factors that determine the mode of delivery of therapeutic preterm labor are mainly maternal factors. Among them, the method of termination of pregnancy is shown in Figure 5.

### 2.3. Learning Method of BP Neural Network

In order to reduce the error between the actual output of the BP network and the expected output to an acceptable range, it is necessary to continuously adjust the weights and thresholds of the BP neural network. Gradient descent is usually used to adjust the weights and node thresholds of the BP neural network. The following will briefly introduce the process of training BP network by gradient descent method [18].

The input vector is

(1) X=x1,x2,…,xn.T

Among them, *n* is the number of input layer units.

Determine the output vector *Y* and the desired output vector *O*, and then the output vector is

(2) Y=y1,y2,…,yq,T

where *q* is the number of output layer units, and then the desired output vector is

(3) O=o1,o2,…,oq.T

Determine the hidden layer output vector *B*.

The output vector of the hidden layer is

(4) B=b1,b2,…,bp.T

Initialize the connection weights from the input layer to the hidden layer.

(5) $$\begin{array}{c} W_{j}={\left[w_{j1},w_{j2},\ldots ,w_{jn}\right]}^{T},j=1,2,\ldots ,p. \end{array}$$

Initialize the connection weights from the hidden layer to the output layer.

(6) $$\begin{array}{c} V_{k}={\left[v_{k1},v_{k2},\ldots ,v_{kp}\right]}^{T},k=1,2,\ldots ,q. \end{array}$$

This process mainly uses the input mode to find the actual output corresponding to it.

Calculate the activation value of each neuron in the hidden layer *s*_*j*_.

(7) $$\begin{array}{c} s_{j}=\sum_{i=1}^{n}w_{ji}x_{i}-\theta_{j},\left(j=1,2,\ldots ,p\right). \end{array}$$

Among them, *w*_*ji*_ represents the weight from the input layer to the hidden layer and *θ*_*j*_ represents the threshold of the hidden layer unit.

The activation function adopts a sigmoid function, that is,

(8) $$\begin{array}{c} f\left(x\right)=\frac{1}{1+\exp\left(-x\right)}. \end{array}$$

Substitute *s*_*j*_ into the activation function to obtain the output value of the hidden layer *j* unit as

(9) bj=fsj=11+exp−∑i=1nwjix+iθj.

Calculate the activation value *s*_*k*_ of the *k*th unit of the output layer.

(10) $$\begin{array}{c} s_{k}=\sum_{j=1}^{p}v_{kj}b_{j}-\theta_{k}. \end{array}$$

In the formula, *θ*_*k*_ is the output layer unit threshold.

Calculate the actual output value of the kth unit of the output layer *y*_*k*_.

(11) $$\begin{array}{c} y_{k}=f\left(s_{k}\right),\left(k=1,2,\ldots ,q\right). \end{array}$$

In the formula, *f*(*x*) is the sigmoid activation function.

The actual input value of the network can be calculated in the previous step. If the difference between the value and the expected value is greater than the specified error, the weights and thresholds of the network are corrected [19]. Since the correction is performed in the reverse direction, it is called error inverse propagation, and the specific process is as follows.

The correction error of the output layer is

(12) $$\begin{array}{c} d_{k}=\left(o_{k}-y_{k}\right)y_{k}\left(1-y_{k}\right),k=1,2,\ldots ,q. \end{array}$$

In the formula, *y*_*k*_ is the actual output and *o*_*k*_ is the desired output.

The correction error of each unit in the hidden layer is

(13) $$\begin{array}{c} e_{j}=\left(\sum_{k=1}^{q}v_{kj}d_{k}\right)b_{j}\left(1-b_{j}\right). \end{array}$$

The correction amount from the output layer to the hidden layer is

(14) $$\begin{array}{c} \Delta v_{kj}=ad_{k}b_{j},\\ \Delta \theta_{k}=ad_{k}. \end{array}$$

In the formula, a is the learning coefficient, *a* > 0.

The correction amount from the hidden layer to the input layer is

(15) $$\begin{array}{c} \Delta w_{ji}=\beta e_{j}x_{i},\\ \Delta \theta_{j}=\beta -e_{j}. \end{array}$$

In the formula, *β* is the learning coefficient and 0 < *β* < 1.

It can be seen here that the correction amount is proportional to the learning coefficient, the error, and the input amount. The learning coefficient is generally set to 0.1∼0.8 [20]. In order to speed up the whole learning process of the BP neural network without causing oscillation, a larger learning coefficient can be used in the early stage of learning and then gradually reduced as the learning process progresses.

## 3. Clinical Comparative Experiment

### 3.1. Experimental Data and Methods

General clinical data were collected from April 2010 to April 2022 in a total of 3470 puerperae who gave birth in the obstetrics department of a people's hospital. Among them, there were 717 cases of preterm birth, and the incidence rate of preterm birth was 20.66%. Among the preterm births, therapeutic preterm birth accounted for 45.19% and primary preterm birth was 54.81%. Severe pre-eclampsia preterm births accounted for 11.16% and spontaneous preterm births accounted for 29.77% of primary preterm births and 16% of total preterm births. Among them, intrauterine infection accounted for 34.19% of the total number of spontaneous premature births, paralyzed uterus and twin pregnancy accounted for 17.95%, and breech presentation accounted for 11.11%. Among the patients, the proportion of therapeutic preterm birth is relatively high, and the main causes of therapeutic preterm birth are early child pain, pregnancy complicated by medical and surgical diseases, multiple pregnancy, and placental factors that lead to early termination of pregnancy. There were 138 cases of spontaneous preterm birth, of which 11 died prematurely, with a mortality rate of 7.97%. Except for one case of twin-to-twin transfusion syndrome death at 36 weeks of gestation (birth weight 600 g), the gestational weeks were mainly concentrated in 28–33 weeks, the average gestational week was 31 weeks, the weight was 570–2030 g, and the average weight was 1394.5 g.

Data processing was performed on SPSS software, and the relationship was considered significant and meaningful when the *p* value was less than 0.05.

### 3.2. Different Causes of Spontaneous Preterm Birth

There are many causes of preterm birth, including intrauterine infection and multiple pregnancy. Moreover, patients admitted to the hospital before 32 weeks and those with preterm birth after 32 weeks usually have different causes, as shown in Table 1.

Intrauterine infection is the main cause of threatened preterm labor at various gestational weeks, and other causes such as uterine malformation and cervical laxity are relatively rare. Cervical cerclage at 14–16 weeks can effectively prevent late miscarriage and premature birth in patients with lax internal os.

As shown in Table 2, the neonatal infection rate of those with premature rupture of membranes was significantly higher than that of those without premature rupture of membranes, which may be due to the communication between the uterine cavity and the external environment of those with ruptured membranes. External bacteria and fungi enter the uterine cavity retrogradely through the reproductive tract, resulting in intrauterine infection of the fetus. It shows that the development of various organs of neonates before 32 weeks is incomplete, the survival rate is low, and there is no clear correlation with whether there is premature rupture of membranes.

### 3.3. Comparison of Early-Onset Severe Preeclampsia Cases at Different Gestational Weeks

As shown in Table 3, there is a significant difference between the delivery cycle and the expectant treatment time between the control group and the observation group, and the *p* value is less than 0.05.

As shown in Figure 6, the cases of different gestational weeks have great differences. Maternal complications and neonatal outcomes improved with increasing gestational age.

### 3.4. Timing of Pregnancy Termination in Early-Onset Severe Preeclampsia

From Table 4, it can be found that most of the early-onset severe eclampsia terminates pregnancy between 33 and 38 weeks.

As shown in Figure 7, with the extension of pregnancy termination weeks, the adverse pregnancy situation will gradually slow down. At less than 32 weeks, pregnant women are more vulnerable, and the fetuses are not fully developed, which can easily lead to complications of pregnant women and asphyxia or death of newborns.

As shown in Figure 8, there are large differences between vaginal and cesarean sections in the presentation of complications and neonatal asphyxia and mortality. After controlling for the confounding effect of gestational age, mode of delivery was associated with different types of preterm birth. The ORMH value was the combined OR value after adjusting for the confounding effect of gestational age, which suggested that the modes of delivery were different among the three groups. After excluding the confounding effect of gestational age, spontaneous preterm vaginal delivery was approximately 83.43 times that of cesarean section, and spontaneous preterm birth was dominated by vaginal delivery. Spontaneous preterm birth is mainly vaginal delivery, with a cesarean delivery rate of only 6.04%, while therapeutic preterm birth is dominated by cesarean delivery, with a cesarean delivery rate as high as 84.91%. There were certain proportions of vaginal delivery and cesarean section in the term delivery group, and the cesarean section rate was 37.83%.

### 3.5. Comparison of Preterm Birth with Severe Preeclampsia and Spontaneous Preterm Birth

After the above experiments, it was found that the week of onset, the timing of termination of pregnancy, and the mode of delivery were all related to maternal complications and neonatal survival. For this, the experimental results are as follows.

As shown in Figure 9, in either case, patients with preterm birth with severe eclampsia had higher morbidity and mortality than spontaneous preterm birth. In cases of less than 32 weeks, there is even maternal death in patients with severe eclampsia.

### 3.6. Comparison between Regular and Irregular Obstetric Inspection Groups

As shown in Table 5, there is no significant difference in age, maximum systolic blood pressure, maximum diastolic blood pressure, and pregnancy age among the three groups of patients, indicating that the grouping in this paper has a good effect.

As shown in Figure 10, regular and irregular obstetric examinations can predict related symptoms in advance and intervene as soon as possible. Observation group 1 was the severe preeclampsia premature delivery group, and observation group 2 was the spontaneous premature delivery group. Not only maternal complications, but also perinatal outcomes can reduce injury. In particular, patients with preterm labor with severe preeclampsia had about 10% fewer related symptoms than the control group.

## 4. Outcome of Severe Preeclampsia Preterm Birth to Spontaneous Preterm Birth

This study showed that the average gestational age was prolonged by 13.63 days for cases within 30 weeks of gestational age. The average gestational week of delivery was 32.76 weeks, and the average gestational week was prolonged by 19.67 days. The average gestational week of delivery was 34.15 days, and the average gestational week was 35.16 days. Due to the small onset of gestational weeks and severe disease in cases with onset within 30 weeks of gestation, although the treatment is actively expected, the effect is limited. The fetus in the 32.76-week case has a certain viability, and the treatment effect is expected to be the best. In the case of 35.16 weeks, when the gestational age after treatment is expected to reach 34 weeks or more, the risk of continuing pregnancy is considered.

Further analysis of the pregnancy outcomes of the three groups showed that the incidence rates of placental abruption, postpartum hemorrhage, liver and kidney dysfunction, and eclampsia in pregnant women with onset before 30 weeks were significantly higher than those with onset after 30 weeks. The perinatal outcomes of pregnant women with onset before 30 weeks were also worse than those after 30 weeks, especially the fetuses delivered by pregnant women with onset at 32 weeks did not have severe ventricular arrhythmias and deaths. It shows that expectant treatment does not significantly increase the occurrence of serious adverse pregnancy outcomes such as ventricular arrhythmia and death. Gestational age at delivery is the most important factor affecting neonatal survival, partly due to the discovery of premature gestational age, which is still less than 34 weeks after expectant treatment. Most cases of early-onset severe preeclampsia are extended beyond 34 weeks of gestation. When the gestational age reached 34 weeks, the incidence of serious complications of maternal childbirth, the incidence of neonatal ventricular arrhythmia, and the probability of perinatal death were significantly reduced. However, this part of the case still increased the gestational age through expectant treatment, and the extended gestational age also brought time for the completion of preparatory work before termination of pregnancy such as promoting fetal lung maturity and at the same time alleviated or improved the condition of the pregnant woman to prepare for delivery. Therefore, patients with early-onset severe preeclampsia should be treated expectantly when both maternal and fetal conditions allow. Of course, during this process, the mother and fetus should be closely monitored, and the pregnancy should be terminated in time when abnormal detection indicators indicate that it is not suitable to continue the pregnancy.

Mode of delivery in severe preeclampsia is based on obstetric indications. However, when the patient's condition is unstable, there are serious complications, the cervix is immature and the fetus cannot be delivered in a short time, and the fetal heart rate is abnormal, the cesarean section can be appropriately relaxed. In this study, cesarean section was the most common method of pregnancy termination for severe preeclampsia, accounting for 92.76%. There was no significant difference in mode of delivery between the early-onset severe preeclampsia group and the late-onset group (*P* > 0.05). Studies have shown that compared with delivery by cesarean section, vaginal delivery has an increased risk of fetal distress and neonatal ventricular asphyxia, which may be related to the stress process that the fetus needs to withstand ischemia and hypoxia during the onset of labor and cesarean section effectively avoids this process. In addition, the high expectations of the newborn and the possible serious complications of the mother during the labor process also make most patients and their families request cesarean section to terminate the pregnancy, in order to reduce the risk to both mother and baby during the vaginal trial production process. In addition, this study found that cesarean section was the most important mode of pregnancy in group *B* (32 weeks < gestational week of termination of pregnancy <34 weeks) and group C (gestational week of termination of pregnancy> 34 weeks), accounting for 92.31, 100.00%. In group A (gestational age of termination of pregnancy <32 weeks), there were 6 cases of vaginal delivery, accounting for 35.29%. Among them, 5 cases of multiparous women suffered from intrauterine distress, umbilical artery diastolic blood flow disappeared, and 1 case of primiparous stillbirth underwent intrauterine water balloon induction of labor. This is related to the poor control of the condition of patients with severe preeclampsia after expectant treatment, the occurrence of intrauterine stillbirth, or the request of the patients and their families to abandon the fetus due to intrauterine distress. There is a traumatic impact of choosing vaginal delivery over avoiding cesarean section on the patient. When giving up the interests of the fetus in patients with severe preeclampsia, the interests of pregnant women should be paid attention to in time.

In this study, the incidence of all complications in the early-onset severe preeclampsia group was higher than that in the late-onset group, but only in the comparison of placental abruption and pleural effusion between the two groups was statistically significant (*P* < 0.05). This study shows that the younger the gestational age, the easier it is to involve various organ systems, and the occurrence of serious complications, especially the occurrence of placental abruption is closely related to the length of expectant treatment. The younger the gestational age and the longer the time to expect treatment, the higher the risk of placental abruption. The higher risk of adverse perinatal outcomes is associated with smaller gestational age at onset, smaller gestational age, and maturation of various organ systems. In addition, the placenta itself has abnormal development in patients with severe preeclampsia, so that the impaired function of the placenta cannot provide sufficient support for the needs of the fetus, which increases the risk of intrauterine growth restriction and intrauterine death. The cesarean section rate of women who gave birth within 32 weeks of gestation was significantly lower than those who gave birth after 32 weeks. It may be related to the smaller gestational age of childbirth, the small expectations of pregnant women and their families for the newborn, and the more consideration of reducing maternal injury and giving up cesarean section. The perinatal mortality rate in the vaginal delivery group was higher than that in the cesarean section group, and the reasons were analyzed. In this study, there were 3 cases of perinatal death cases of vaginal delivery before 32 weeks of gestation, and all 3 cases were delivered before 31 weeks of gestation. Among them, 1 case was delivered at 26 weeks, and the gestational age of delivery was too small, and the prognosis was poor regardless of whether cesarean section or vaginal delivery was selected. However, there was no significant difference in the incidence of maternal complications and neonatal ventricular arrhythmia between the cesarean section group and the vaginal delivery group, so the effect of the two delivery methods on pregnancy outcomes was not obvious when the pregnancy was terminated within 32 weeks. Vaginal delivery is possible under close supervision when maternal and fetal conditions permit.

Due to individual differences in patients, there is currently no unified treatment plan for cases of expectant treatment. Hospitalized patients should be exercised appropriately, and absolute bed rest should be avoided, which increases the risk of bed rest-related venous thrombosis. Fetal ECG monitoring at least once a day and dynamic monitoring of laboratory-related examination items (including: blood routine, urine routine, liver and kidney function, and coagulation function) at least once a week. Dynamic ultrasound monitoring of intrauterine growth and amniotic fluid can reduce the incidence of perinatal death.

## 5. Conclusions

Both severe preeclampsia preterm birth and spontaneous preterm birth have a greater impact on pregnant women and neonates. This paper focuses on the analysis of the clinical differences between the two. After research, the conclusions are as follows:

1. Cases of early-onset severe preeclampsia at different gestational weeks. With the retreat of gestational weeks, complications, and neonatal mortality, and asphyxia rates have decreased, so for severe preeclampsia cases, the timing of pregnancy termination should be delayed as much as possible.
2. Different delivery methods have a greater impact on preterm patients. Among them, the complication of severe preeclampsia in the vaginal delivery method is less than that of the cesarean section, but the neonatal mortality rate of the vaginal delivery method is higher than that of the cesarean section.
3. Compared with spontaneous abortion, preterm women with severe preeclampsia have higher complications and neonatal mortality. Therefore, pregnant women with premature birth should pay attention to regular and regular inspections.

However, there are not many samples in this study, so further research with large clinical samples is needed. At the same time, due to the limited sample size and the temporary unconditional long-term follow-up of all newborns, the impact of cesarean section on the late prognosis of premature infants cannot be clearly determined, so this aspect will be further studied in the follow-up research.

## Figures and Tables

**Figure 1:** Prediction of preterm birth.

**Figure 2:** Treatment of preterm birth.

**Figure 3:** Effects of severe preeclampsia on pregnant women and fetuses.

**Figure 4:** Symptoms of pregnant women with severe preeclampsia.

**Figure 5:** Methods of termination of pregnancy.

**Figure 6:** Comparative analysis of cases at different gestational weeks. (a) Complication comparison. (b) Comparison of perinatal outcomes.

**Figure 7:** Trends in adverse pregnancy outcomes.

**Figure 8:** Comparison of outcomes of different delivery methods. (a) Complications. (b) Neonatal asphyxia or death.

**Figure 9:** Preterm birth in severe preeclampsia compared to spontaneous preterm birth.

**Figure 10:** Comparison of regular and irregular obstetric inspection groups. (a) Comparison of maternal complications. (b) Perinatal prognosis

**Table 1:** Etiological analysis of preterm birth.

Grouping	Admission before 32 weeks (%)	Admission after 32 weeks	Svm (%)
Intrauterine infection	52	27%	34
Multiple pregnancy	21	16%	18
Breech (except twins)	24	6%	11
Scarred uterus	21	17%	18
Polyhydramnios	6	11%	9
Reproductive tract abnormalities	3	10%	8
Cervical laxity	9	0	3

**Table 2:** Comparison of tire protection time.

Grouping	Proportion (%)	Tire protection time (days)
Breech (except twins)	17.07	5.13±3.15
Intrauterine infection	26.83	2.98±1.18
Multiple pregnancy	24.39	16.8±16.15
Scarred uterus	21.95	13±12.97
Polyhydramnios	9.76	7.95±5.15

**Table 3:** Comparison of time to termination of pregnancy and time to expectant treatment.

	Gestational age (weeks)	Expected treatment time (d)
Observation group 1	32.13±2.15	13.23±3.15
Observation group 2	34.98±1.18	19.98±6.18
Control group	35.85± 1.64	11.3±6.15
*P*	<0.001	<0.001

**Table 4:** Composition ratio of time to termination of pregnancy in cases of early-onset severe preeclampsia.

Termination of pregnancy gestational weeks (weeks)	Proportion (%)
<28	2
28–30	5
31–32	8
33–34	34
35–36	28
37–38	20
>38	3

**Table 5:** Basic information.

	Observation group 1	Observation group 2	Control group	*P*
Age (years)	28.65 ± 4.97	32.65 ± 4.67	30.63 ± 5.67	0.003
Maximum systolic blood pressure (mmHg)	157.36 ± 17.46	159.34 ± 16.76	165.39 ± 22.13	<0.001
Maximum diastolic blood pressure (mmHg)	106.65 ± 13.21	111.61 ± 12.93	110.59 ± 12.03	0.003
Urine protein quantification	4.73 ± 4.27	5.93 ± 5.27	5.06 ± 5.11	0.231
Earliest gestational age	32.19 ± 3.97	35.19 ± 5.07	32.19 ± 4.93	0.510
Gestational age	36.54 ± 2.36	38.54 ± 3.36	34.88 ± 2.37	<0.001
Primipara	76.65%	60.35%	65%	<0.001

## Data Availability

Data sharing is not applicable to this article as no datasets were generated or analyzed during the current study.
